The article "Clinical Characteristics, Treatment, and Visual Prognosis in Pediatric Endophthalmitis: A 232-Case Retrospective Study" was retracted in 2023. Reasons: signs of a paper mill; suspected computer-generated content; unreliable results or conclusions; lack of ethics approval or compliance.

# Clinical Characteristics, Treatment, and Visual Prognosis in Pediatric Endophthalmitis: A 232-Case Retrospective Study

**DOI:** 10.1155/2022/8523747

**Published:** 2022-05-09

**Authors:** Fantao Lv, Haiyan Wang, Dawei Zhang, Shengwei Wu

**Affiliations:** Department of Ophthalmology, Beijing Luhe Hospital Capital Medical University, Beijing 101199, China

## Abstract

**Objective:**

In infective endophthalmitis, once the patient's vision is seriously damaged, the damage to children's vision is particularly serious. The main purpose of this study is to investigate the etiology, epidemiology, treatment, and visual prognosis of children's endophthalmitis and to conduct an in-depth analysis. *Study Design*. This study collected case data from the Beijing Tongren Hospital Capital Medical University in the period from January 1, 2002 to January 1, 2018. The basic conditions for inclusion in the collection range were patients who were less than or equal to 14 years old and had a history of infectious endophthalmitis. A retrospective study and analysis of etiology, epidemiology, treatment, and visual prognosis were performed. Kappa and Chi square test were used for statistical analysis.

**Results:**

A total of 232 cases were collected, with an average age of 6.33 ± 2.89 years (range 8months to 14 years). The most common etiologies were ocular trauma (93.5%) and previous ocular surgery (5.2%). Overall, 81 samples were sent to the microbiology department for direct smear and culture, from which 21 organisms were isolated. 28 cases (39.5%) were culture-positive. The most organism was Gram-positive organisms. In treatment, the proportion of PPV use combined with silicone oil filling had increased gradually in three phases, while the other treatments were almost decreased or nearly similar. The final visual result is 22 (9.5) in 20/200 or better, 65 (28.0) in CF-20/200, 38 (16.4) in hand move (HM), 27 (11.6) in light perception (LP), 21 (9.1) in no light perception (NLP), and 59 (25.4) did not match (NM).

**Conclusion:**

Penetrating ocular trauma is the most common cause of infectious endophthalmitis in children. The detection rate of microorganisms is low and helpless for the treatment. In this study, it was found that despite the aggressive treatments such as antibacterial and vitrectomy, the ultimate improvement in vision was highly undesirable.

## 1. Introduction

Infectious endophthalmitis is a serious blinding eye disease caused by the microbial infection of intraocular tissue. If the diagnosis and treatment are delayed or improperly treated, it can lead to irreversible vision loss. According to the transmission route of infection source, it can be divided into exogenous and endogenous: Exogenous is mostly caused by trauma and surgery, while endogenous is caused by bacterial blood flow to intraocular infection. Ocular trauma is the first pathogenic factor of infectious endophthalmitis in China. Outbreak of infectious endophthalmitis in children is rare, but it can cause severe damage to vision and even blindness in many cases. Endophthalmitis in the pediatric population could not only bring children the suffering of disease, but also create a serious economic burden for the family and society. In China, the incidence of pediatric endophthalmitis after open-globe injuries ranges from 9.7% to 20.6% [1, 2], much higher than that in developed countries reported in 2.5% [3] to 3.5% [4]. Unlike adults, it is difficult for children to recognize or verbalize clearly their symptoms, such as decreased visual acuity, photophobia, and pain, which is a challenge to early diagnosis and treatment in the pediatric age group [5].

Infectious endophthalmitis is acknowledged as an important cause of blindness all over the world. However, there is little attention and research devoted to pediatric endophthalmitis unlike the adult population [6]. Some related previous reported samples are consequently sparse. Weinstein et al. published 8 cases of culture-positive pediatric endophthalmitis from 1965 to 1979 [3]; Thordsen et al. [6] reported 16 cases of pediatric endophthalmitis in 2008, Al-Rashaed et al. [4] reported 49 cases, and Zhang et al. [7] reported 271 cases in 2016. However, the number of cases is small in these researches, and the research is not timely. Thus, we reviewed the medical records of all children 14 years and younger with infectious endophthalmitis treated at Beijing Tongren Hospital between January 1, 2002, and February 21, which has a total of 232 cases. For each case, we obtained the children's age, sex, type of injury, initial visual acuity, vitreous culture results, treatment regimen, and visual outcomes. In this retrospective study, we provide detailed epidemiological data on the etiology, epidemiology, treatment, and prognosis of childhood infectious endophthalmitis in a single institution in China over the past 16 years. We hope this will facilitate prompt diagnosis and treatment of endophthalmitis in children.

## 2. Materials and Methods

This retrospective study included 232 cases, which we reviewed of all children 14 years and younger with infectious endophthalmitis treated at Beijing Tongren Hospital between January 1, 2002, and January 1, 2002.This study was approved by the same ethics committee of the same institution. The diagnosis of infectious endophthalmitis was based on patient histories, ophthalmic examinations, and supplementary examinations. The cases were divided into post-traumatic group (*n* = 271), postoperative group (*n* = 12), and endogenous group (*n* = 3) with regard to type of injury. In addition, we divided the cases into 3 periods according to the year in which the case occurred (2002-2006, named Group 1; 2007-2012, named Group 2; and 2013-2017, named Group 3) and compared the characteristics of the cases among these 3 groups. Our objective was to provide more confirmatory data and evidence in terms of the cause, treatment, and prognosis of pediatric endophthalmitis.

For each case, we recorded the patients' age, sex, precipitating event, type of ocular trauma, time from injury to first presentation and treatment, initial visual acuity, results of slit-lamp examination, vitreous culture results, therapeutic methods, follow-up treatment out of the hospital, and final visual acuity.

Vitreous and aqueous samples were obtained by needle aspiration or vitrectomy and sent to the microbiology department for direct smear and culture. All patients received immediate intravenous and topical antibiotics as required, and further drug therapy was guided by the culture results. Pars plana vitrectomy (PPV) should be considered if there is a significant deterioration within 24 hours, or if there is no response to treatment within 48 hours after the first intravitreal antibiotic injection, and intravitreal injection with a sensitive antibiotic may also be used. Early PPV is required in the presence of intraocular foreign bodies, traumatic retinal detachment, and lens dislocation [8].

Statistical analyses were performed with SPSS software (SPSS 22.0). Continuous variables were expressed as mean ± standard deviation (SD). Kappa test was used to assess the uniformity between the direct smear results and culture results of the specimen. In addition, Pearson chi-square tests were used to determine the differences in the proportions of treatment methods and final VA among 3 periods. *P* values of <0.05 were considered statistically significant.

## 3. Results

### 3.1. Clinical Characteristics

On the whole, 232 eyes of 232 children were enrolled in our study (167 males [72.0%] and 65 females [28.9%]), with a mean age of 6.33 ± 2.89 years (range, 1 year to 14 years). The distributions of the patient ages and onset years are illustrated in Figure 1. From these data, we could note that the age of peak incidence was 3–6 years, more specifically 4–5 years. Of the 232 eyes in this study, 133 were right eyes and 199 were left eyes.

The most common etiology of pediatric infectious endophthalmitis is ocular trauma, accounting for 217 (93.5%) of 232 cases. Postoperative endophthalmitis developed in 12(5.2%) of all case, which followed cataract surgery in 9 cases, and glaucoma trabeculectomy in 3 cases. The remaining cases of PTE was resulted from endogenous. A total of 217 cases were related to ocular trauma; disposable syringe (44 cases, 19.0%) was the most common source of injuries, followed by woodware such as plant branch, sawdust, and wood brick. The remaining sources are illustrated in Figure 2.

The number of cases fluctuated from 2002 to 2017, but the overall trend was downward, which dropped from 22 in 2002 to 7 in 2017. The climax was 26 in 2009 (Figure 3).

The time window from onset to diagnosis of endophthalmitis was within 1 week in 84 cases, 1-2 weeks in 60 cases, 2-3 weeks in 46 cases, 3-4 weeks in 19 cases, and more than 4 weeks in 23 cases. (Table 1).

Table 2 shows the number of cases in the most common age group every year from 2002 to 2017. We could figure out that the most one was 6 in 2007 which was belonged to 6<age ≤7 and in 2009 which was belonged to 3<age ≤4.

In the 5-year cluster data of the etiologies, the top three were infusion needle, the other types of disposable syringe, and the woodware in Group 1; the infusion needle, the woodware, and metal objects in Group 2; and the woodware, the scissors, and the other types of disposable syringe in Group 3. On the whole, the most common 3 etiologies were the infusion needle, the woodware, and the other types of disposable syringe (Figure 4) Further, we extracted the posttraumatic cases to analyze and found that the percentage of the infusion needle reduced gradually, while the percentage of the woodware increased as time went on (Figure 5).

81 cases were sent to the microbiology department for direct smear and culture, from which 21 organisms was isolated. 28 cases (39.5%) were culture-positive. The most organism was Gram-positive organisms, and only 1 case isolated *Geotrichum candidum*. Considering the number of cases with causative organisms was too small, we did not think these data have statistical significance.

### 3.2. Treatment

All children received immediate treatment with intravenous and topical antibiotics as soon as they visited our hospital. Vancomycin and ceftazidime or amphotericin B were used as empirical intravitreal antibiotics, part of cases depending on the intraoperative direct smear results. 7 cases (3.0%) were treated with only infusion; 1 case (0.4%) with intraocular antibiotics. Pars plana vitrectomy (PPV) as the single method of pediatric infectious endophthalmitis (PIE) treatment was applied in some children with serious vitreous inflammation (36 cases, 15.5%). 18 cases (7.8%) were treated with PPV and intravitreal injections of antibiotics. 146 eyes (62.9%) underwent vitrectomy combined with silicone oil filling, and 13 cases (5.6%) underwent combined with gas filling. 5 eyes (2.2%) were enucleated or eviscerated due to serious intraocular inflammation that did not respond to treatment. The proportion of PPV use combined with silicone oil filling had increased gradually in three phases, while the other treatments were almost decreased or nearly similar (Table 3 and Figure 6).

### 3.3. Visual Prognosis

The final VA is summarized in Table 3. The mean follow-up time was 19.1 months (range 7 months to 5 years). The final VAs of 64 cases were not obtained because they were too small or their condition were too complex to have visual examinations. There were only 21 eyes (9.1%) with a final VA of 20/200 or better, while 18 patients (7.8%) had a final VA without light perception. In this study, we did not find any statistically significant association between the time of onset and the prognosis of endophthalmitis.

Despite of active management with antibiotics and surgery, visual impairment was common in most of cases. To determine whether visual acuity could be improved as time went on, a comparison of final VA in different periods is illustrated in Table 4.

We could conclude that the differences were statistically significant (*P* < 0.05) in 3 groups which had a final VA of NLP after comparison. After a pairwise comparison, the proportion of NLP in Group 2 was higher than in Group 1, which had a statistical significance (adjust *P* < 0.05). The comparison between Groups 3 and 1, as well as Groups 2 and 1, had no statistical significance in NLP (adjust *P* > 0.05). The differences in the final VA of 20/200 or better among 3 groups had a statistical significance (*P* < 0.05). Group 1 had more patients with final VA of 20/200 or better than Group 3 (adjust *P* < 0.05), while there was no difference between Groups 2 and 1, as well as Groups 1 and 2 by contrast (adjust *P* > 0.05).

## 4. Discussion

Pediatric endophthalmitis is a rare but serious disease often associated with irreversible loss of vision. In our study, penetrating ocular trauma was the most common leading cause of pediatric endophthalmitis, whereas the endogenous infections are the least common cause. In the developed country, toys with sharp ware or articles of everyday use were the most common etiologies in contrast to disposable syringes and woodware in developing countries. It is worth mentioning that with the time went on, we could see a decline in proportion of disposable syringes causing PTE which may thank to the improving standardized management of medical supplies and ubiquitous compulsory education in rural or some other less developed areas.

Surgery was the second common cause especially in cataract and glaucoma-filtering surgeries because congenital cataracts and congenital glaucoma were found to have the highest incidences in children. Risk factors of cataract surgery included vitreous loss, inadequate disinfection, and leakage of the incision. Glaucoma-filtering-surgery-related endophthalmitis had a close relationship with filtering blebs. In general, the window time of endophthalmitis caused by glaucoma surgery was often longer than cataract surgery. With the innovation of the operation itself and postoperative nursing technology, the incidence was on decline. Nevertheless, some study reported that postoperative endophthalmitis accounting for majority (72%) which was quite different from ours (5.2%).

Recently, pars plana vitrectomy in treatment of PIE had played a key role. It had widely recognized the timely PPV as the management in serious PTE patients could control the disease effectively and have a better visual prognosis [9]. Patients treated with vitrectomy and intravitreal antibiotics had better visual effects than those treated with antibiotics alone as reported by Al-Rashaed et al. [4]. The final VA with NLP in children treated with PPV accounted for 6.1% that obviously less than those treated with antibiotics alone, 42.8%.16.9% patients had a final VA of counting figures after PPV. These results indicated that vitrectomy was more effective for children with endophthalmitis. What's more, in the five-year grouping, it was found that vitrectomy combined with silicone oil filling had become the main surgical method and its proportion was increasing gradually. Thus, PPV could be thought of a preferred treatment of PIE.

In our study, however, there were several limitations. The data are from a single tertiary referral center, and initial diagnosis and treatment are performed by different doctors in different medical institutions, which may not be representative of those found in other settings. In this series of studies, the prognosis of endophthalmitis after eye surgery was better than those of other causes. This result may be confined by the small sample size and the pediatric population so it can not apply to all age groups.

In summary, penetrating ocular trauma is considered to be the most common cause of pediatric endophthalmitis in China, and disposable syringe is the most common etiology, while wood products and knives should be paid more attention in recent years. By comparing the data of three periods, the most common etiology had changed slightly, which may have an association with the improvement of living standards and medical care.

In addition to essentially having enough antibiotics in a timely manner, PPV should be taken into consideration. In spite of aggressive management with antibiotics and PPV, PTE in children generally has a poor visual prognosis.

In this retrospective study, we provided detailed epidemiological data on the etiology, epidemiology, treatment, and prognosis of infectious endophthalmitis in children from a single institution in China over the past 16 years. We hope that this will be helpful to the timely diagnosis and treatment of pediatric endophthalmitis.

## 5. Conclusion

Penetrating ocular trauma is the most common cause of infectious endophthalmitis in children. The most common cause of penetration has gradually changed from syringes to wood products and knives. The detection rate of microorganisms is low and is useless for treatment. In this study, it was found that PPV + oil has gradually become the preferred treatment for children with severe endophthalmitis, and despite the aggressive treatments, the ultimate improvement in vision was highly undesirable.

## Figures and Tables

**Figure 1:** Age's distribution.

**Figure 2:** Percentage of cases caused by different types of ocular trauma.

**Figure 3:** General trends of incidence over the past 15 years.

**Figure 4:** The percentage of the etiology in every-5-year groups.

**Figure 5:** Trend changes in different periods of the most common etiologies.

**Figure 6:** Change trend of the operation in every-5-year groups.

**Table 1:** The distribution of the final VA cases in operation time.

The time window from onset to operation	Final VA, *n* (%)						
	NA	NLP	LP	HM	CF-20/200	20/200 or better	Total
In 1 week	18 (21.4)	4 (4.8)	8 (9.5)	16 (19.0)	29 (33.7)	9 (10.7)	84 (36.2)
1 week to 2 weeks	25 (41.7)	8 (13.3)	4 (6.7)	8 (13.1)	11 (18.3)	4 (6.7)	60 (25.9)
2 weeks to 3 weeks	11 (23.9)	2 (4.3)	11 (23.9)	8 (17.4)	12 (26.1)	2 (4.3)	46 (19.8)
3 weeks to 4 weeks	3 (15.8)	1 (5.3)	1 (5.3)	6 (31.6)	6 (31.6)	2 (10.5)	19 (8.2)
More than 4 weeks	7 (30.4)	3 (13.0)	1 (4.3)	2 (8.7)	6 (26.1)	4 (17.4)	23 (9.9)
Total	64 (27.6)	18 (7.8)	25 (10.8)	40 (17.3)	64 (27.6)	21 (9.1)	232

**Table 2:** The distribution of patient's age and onset year.

Age	2002	2003	2004	2005	2006	2007	2008	2009	2010	2011	2012	2013	2014	2015	2016	2017	Total
A <1	1	0	0	0	0	0	0	0	1	0	1	0	0	0	0	0	3
1 ≤ A ≤2	2	0	0	1	0	3	2	1	1	0	0	0	1	0	1	0	12
2 ≤ A ≤3	1	1	2	1	2	2	3	2	0	2	0	2	1	0	1	1	21
3 ≤ A ≤ 4	5	3	1	1	2	2	3	6	4	2	1	2	0	1	1	0	34
4 ≤ A ≤ 5	2	4	0	1	4	1	5	4	4	2	4	1	2	0	2	0	36
5 ≤ A ≤ 6	2	0	1	0	3	4	4	2	2	1	2	0	1	1	1	0	24
6 ≤ A ≤7	0	1	0	1	1	6	3	2	1	0	3	1	2	3	1	1	26
7 ≤ A ≤ 8	2	3	2	3	1	0	1	1	1	0	3	0	0	1	1	2	21
8 ≤ A ≤ 9	2	0	2	1	1	4	1	3	2	0	0	1	0	2	0	1	20
9 ≤ A ≤ 10	3	3	0	0	1	2	0	1	0	0	0	0	0	1	0	0	11
10 ≤ A ≤ 11	1	1	1	1	0	0	0	0	1	3	0	1	0	1	0	1	11
11 ≤ A ≤ 12	0	1	0	1	0	1	0	1	1	0	0	0	0	0	0	1	6
12 ≤ A ≤ 13	0	1	0	0	0	0	0	1	0	0	0	0	0	0	0	0	2
13 ≤ A ≤ 14	1	0	0	0	0	0	0	2	0	0	1	0	1	0	0	0	5
Total	22	18	9	11	15	25	22	26	18	10	15	8	8	10	8	7	232

**Table 3:** Relationship between operative method and final VA.

Operative method	Final VA, *n* (%)						Total
	EE	NLP	LP	HM	CF-20/200	20/200 or better	
INA	3 (42.9)	3 (42.9)	0 (0)	0 (0)	1 (14.2)	0 (0)	7 (3.0)
PPV	8 (21.6)	0 (0)	4 (10.8)	8 (21.6)	14 (37.8)	3 (8.1)	37 (15.9)
PPV + INA	5 (44.4)	1 (5.6)	3 (16.7)	2 (11.1)	2 (11.1)	5 (27.8)	18 (7.8)
PPV + oil	40 (27.6)	12 (8.3)	19 (13.1)	24 (16.6)	39 (26.9)	11 (7.6)	145 (62.5)
PPV + gas	1 (7.7)	0 (0)	0 (0)	4 (30.8)	7 (53.8)	1 (7.7)	13 (5.6)
Enucleated	0 (0)	5 (100)	0 (0)	0 (0)	0 (0)	0 (0)	5 (2.2)
Inv	2 (28.6)	0 (0)	1 (14.2)	0 (0)	2 (28.6)	2 (28.6)	7 (3.0)
Total	59 (25.4)	21 (91)	27 (11.6)	38 (16.4)	65 (28.0)	22 (9.5)	232

∗INA: intravitreal antibiotic injection; PPV: pars plana vitrectomy; PPV + oil: pars plana vitrectomy combined with silicone oil filling; PPV + gas: pars plana vitrectomy combined with gas filling; Inv: intravenous injection; VA: visual acuity; EE: enucleated or eviscerated; NLP: no light perception; LP: light perception; HM: hand motions; CF: counting fingers.

**Table 4:** The comparison of the every-5-year series in the final VA.

The every-5 year series	Final VA, *n* (%)						Total
	EE	NLP	LP	HM	CF-20/200	20/200 or better	
1	3 (4.0)	7 (5.3)	14 (18.7)	19 (25.3)	15 (20.0)	17 (22.7)	75 (33.3)
2	16 (15.8)	10 (9.9)	14 (13.9)	20 (19.8)	14 (13.9)	27 (26.7)	101 (44.9)
3	7 (14.3)	8 (16.3)	8 (16.3)	8 (16.3)	2 (4.1)	16 (32.7)	49 (21.8)
*χ* ^2^	6.362	1.739	0.744	1.586	0.357	1.512	
*Ρ*	0.042	0.419	0.689	0.453	0.934^∗^	0.470	

∗Means using the Fisher's exact probability method.

## Data Availability

The data used to support the findings of this study are available from the corresponding author upon request.
